This article has been retracted.

# Circular RNA hsa_circ_0000517 modulates hepatocellular carcinoma advancement via the miR-326/SMAD6 axis

**DOI:** 10.1186/s12935-020-01447-w

**Published:** 2020-08-03

**Authors:** Shuwei He, Zhengwu Guo, Qian Kang, Xu Wang, Xingmin Han

**Affiliations:** 1 Department of Nuclear Medicine, The First Affiliated Hospital of Zhengzhou University, Zhengzhou, Henan 450000 China; 2 Henan Medical Key Laboratory of Molecular Imaging, No. 1 Jianshe East Road, Zhengzhou, Henan 450000 China

**Keywords:** HCC, hsa_circ_0000517, miR-326, SMAD6

## Abstract

**Background:**

Hepatocellular carcinoma (HCC) is the most common malignant heterogeneous disease in primary liver tumors. Circular RNA hsa_circ_0000517 (hsa_circ_0000517) is connected with HCC prognosis. Nevertheless, there are few studies on the role and mechanism of hsa_circ_0000517 in HCC.

**Methods:**

Expression of hsa_circ_0000517, miR-326, and SMAD family member 6 (SMAD6) was detected by quantitative real-time polymerase chain reaction (qRT-PCR). Cell viability, colony formation, cell cycle, migration, and invasion were determined though Cell Counting Kit-8 (CCK-8), colony formation, flow cytometry, wound healing, or transwell assays. Protein levels of Cyclin D1, matrix metalloproteinase-2 (MMP2), matrix metalloproteinase-9 (MMP9), SMAD6, and proliferating cell nuclear antigen (PCNA) were examined with western blot analysis. The relationship between hsa_circ_0000517 or SMAD6 and miR-326 was determined via dual-luciferase reporter and RNA immunoprecipitation (RIP) assays. The role of hsa_circ_0000517 in vivo was confirmed via xenograft assay.

**Results:**

Hsa_circ_0000517 and SMAD6 were up-regulated while miR-326 was down-regulated in HCC tissues and cells. Hsa_circ_0000517 down-regulation repressed cell proliferation, colony formation, migration, and invasion, and induced cell cycle arrest in HCC cells in vitro, and constrained tumor growth in vivo. Notably, hsa_circ_0000517 regulated SMAD6 expression via acting as a competing endogenous RNA (ceRNA) for miR-326. And the repressive influence on malignant behaviors of HCC cells mediated by hsa_circ_0000517 inhibition was reversed by miR-326 inhibitors. Moreover, SMAD6 elevation overturned the inhibitory impacts of miR-326 mimics on malignant behaviors of HCC cells.

**Conclusions:**

Hsa_circ_0000517 depletion repressed HCC advancement via regulating the miR-326/SMAD6 axis.

## Highlights

1. Hsa_circ_0000517 expression was increased in HCC tissues and cells.
2. Inhibition of hsa_circ_0000517 repressed HCC progression.
3. Hsa_circ_0000517 acted as a ceRNA for miR-326.
4. SMAD6 was a target for miR-326.
5. Hsa_circ_0000517 regulated SMAD6 expression via miR-326.

## Background

Hepatocellular carcinoma (HCC), the most common malignant heterogeneous disease in primary liver tumors, ranks fourth among cancer-related causes of death [1]. At present, the treatment of HCC mainly includes surgery, radio-therapy, or chemo-therapy [2, 3]. Despite advances in the diagnosis of HCC, only 30–40% of patients can be treated with surgery [4]. The main reason for losing surgical treatment is because most patients are diagnosed at an advanced stage [5, 6]. However, most HCC patients have metastases and relapses within 5 years after undergoing surgical treatment [7, 8]. In consequence, it is vital to survey the mechanisms related to HCC progression for developing new diagnostic biomarkers and treatment strategies.

Circular RNAs (circRNA) are a special type of non-coding RNAs with a covalently closed continuous circular structure [9]. They are abundant, stable, and conserved, and are usually expressed at a particular developmental stage or in specific tissues [10]. Improving evidence has demonstrated that circRNAs can control gene expression by regulating RNA-binding proteins by working as a competing endogenous RNA (ceRNA) for microRNAs (miRNA) [11]. Recently, many circRNAs were revealed to be involved in tumor advancement [12]. Circular RNA hsa_circ_0000517 (hsa_circ_0000517) is transcribed from the ribonuclease P RNA component H1 (RPPH1) gene on chromosome14:20811404-20811492. Moreover, hsa_circ_0000517 acted as a novel promising biomarker for the prediction of HCC prognosis [13]. Notwithstanding, the function and mechanism of hsa_circ_0000517 in cancer are rarely reported.

MiRNAs modulate the expression of target genes after transcription [14]. They exert vital roles in a verity of biological processes, such as developmental, proliferation, metabolism, and differentiation [15]. MiRNAs serve as tumor suppressors or oncogenes to regulate tumor progression and metastasis [16]. For instance, miR-203 accelerated tumor growth and cell stemness in ER-positive breast, while it repressed cancer cell growth in gastric cancer [17, 18]. It was reported that microRNA-326 (miR-326) down-regulation was connected with gastric cancer poor prognosis [19]. MiR-326 was disclosed to be implicated in the development of diverse tumors, such as endometrial cancer [20], colorectal cancer [21], and lung cancer [22]. Also, miR-326 mediated cell apoptosis, invasion, and proliferation in HCC [23]. However, the molecular mechanisms of miR-326 in HCC need to be further studied.

SMAD family member 6 (SMAD6) is a vital feedback suppressive modulator of bone morphogenetic protein (BMP)/SMAD signaling [24]. Imbalance of BMP signaling in developmental syndromes can accelerate the progression of diseases, including cancers [25]. In a zebrafish xenograft model, SMAD6 could determine BMP-mediated breast cancer cell invasion behavior [26]. SMAD6 negatively modulated PIAS3-mediated suppression, which accelerated cell growth and stem-like initiation in glioma cells [27]. Also, BRG1 accelerated SMAD6 expression in HCC cells, which could facilitate cancer cell proliferation [28]. However, the molecular mechanisms of SMAD6 in the progression of HCC have not been fully elucidated.

Hence, we explored the role of hsa_circ_0000517 in HCC. Moreover, we also surveyed the molecular mechanism of the hsa_circ_0000517/miR-326/SMAD6 axis in HCC cells.

## Materials and methods

### Patients and specimens

All experimental protocols in this research were ratified by the Ethics Committee of the First Affiliated Hospital of Zhengzhou University. 50 paired HCC tissues and adjoining normal tissues were obtained from HCC patients who underwent surgery at the First Affiliated Hospital of Zhengzhou University. The clinicopathological parameters of patients with HCC were exhibited in Table 1. The criteria for inclusion in our sample were: patients with complete survival data and no chemotherapy or radiotherapy before surgery. The patients were followed up for 5 years and no patients were lost to follow-up during this period. Informed consent was signed by the each participant prior to surgery.

**Table 1:** Correlation between hsa_circ_0000517 expression and clinicopathological parameters of hepatocellular carcinoma patients (n = 50)

Clinical feature	n	hsa_circ_0000517		*P*-value
		High	Low	
Age				0.5688
≥ 60	28	15	13	
< 60	22	10	12	
Gender				0.5443
Man	34	18	16	
Woman	16	7	9	
Tumor size				*< 0.0001*
≥ 5 cm	30	22	8	
< 5 cm	20	3	17	
TNM state				*0.0016*
III	29	20	9	
I + II	21	5	16	
Lymph node metastasis				*0.0039*
Negative	30	20	10	
Positive	20	5	15	

The italics *P* values had significant differences

### Cell culture and transfection

Hepatic epithelial cells THLE-2 and HCC cell lines (HCCLM3, Huh7, and MHCC97-H) were purchased from BeNa Culture Collection (Suzhou, China). All cells were kept in an incubator with 5% CO_2_ at 37 °C and cultured in Roswell Park Memorial Institute (RPMI) 1640 medium (Sigma, Louis, Missouri, MO, USA) complemented with fetal bovine serum (FBS, 10%, HyClone, Logan, UT, USA), streptomycin (100 μg/mL, Sigma), and penicillin (100 U/mL, Sigma).

Small interference RNA targeting hsa_circ_0000517 (si-hsa_circ_0000517#1 and si-hsa_circ_0000517#2) and negative control (si-NC) were obtained from GenePharma (Shanghai, China). MiR-326 mimics and inhibitors (miR-326 and anti-miR-326) and their negative controls (NC and anti-NC) were procured from GenePharma. The sequence of hsa_circ_0000517 or SMAD6 was cloned into the pCD5-ciR vector (circ-NC) (Greenseed Biotech, Guangzhou, China) or pcDNA3.1 vector (vector) (Invitrogen, Carlsbad, CA, USA) to construct the overexpression vectors for hsa_circ_0000517 and SMAD6, respectively. When the confluence reached 80%, HCC cells were transiently transfected with the designated plasmids or oligonucleotides using Lipofectamine 3000 reagent (Life Technologies, Grand Island, NY, USA).

### Quantitative real-time polymerase chain reaction (qRT-PCR)

Total RNA of specimens, HCC xenograft tissues, and cells was extracted through the TRIzol reagent (Life Technologies). For RNase R digestion, total RNA of HCC cells was treated with RNase R (3 U/μg, Epicentre Technologies, Madison, WI, USA) at 37 °C for 15 min. Total RNA (1 μg) was reverse transcribed using the PrimeScript RT reagent Kit (Takara, Dalian, China) or miRNA First-Strand Synthesis Kit (Takara) to obtain the complementary DNA for hsa_circ_0000517, RPPH1, SMAD6, and miR-326. QRT-PCR was conducted through the SYBR Premix Ex Taq (Takara). The 2^−ΔΔCt^ method was employed to figure the expression of hsa_circ_0000517, RPPH1, SMAD6, and miR-326, and Glyceraldehyde-3-phosphate dehydrogenase (GAPDH) or U6 small nuclear RNA (snRNA) was served as an internal control. The sequence of the primers were used in this research as below: GAPDH: (F: 5′-GACTCCACTCACGGCAAATTCA-3′ and R: 5′-TCGCTCCTGGAAGATGGTGAT-3′); hsa_circ_0000517: (F: 5′-GGGAGGTGAGTTCCCAGAGA-3′ and R: 5′-TGGCCCTAGTCTCAGACCTC-3′); RPPH1: (F: 5′-CGAGCTGAGTGCGTCCTGTC-3′ and R: 5′-TCGCTGGCCGTGAGTCTGT-3′); SMAD6: (F: 5′-GCTACCAACTCCCTCATCACT-3′ and R: 5′-CGTCGGGGAGTTGACGAAGAT-3′); U6 snRNA (F: 5′-GCTCGCTTCGGCAGCACA-3′ and R: 5′-GAGGTATTCGCACCAGAGGA-3′), and miR-326 (F: 5′-GGCGCCCAGAUAAUGCG-3′ and R: 5′-CGTGCAGGGTCCGAGGTC-3′).

### Cell Counting Kit-8 (CCK-8) assay

After transfection with the designated plasmids or oligonucleotides, the HCCLM3 and Huh7 cells (5 × 10^3^) were cultured in RPMI 1640 medium for 48 h. Next, the CCK-8 reagent (10 μL, Dojindo, Tokyo, Japan) was added into each well and incubated for 2 h. The color reaction at 450 nm was analyzed through the Microplate Absorbance Reader (Bio-Rad Labs., Richmond, CA, USA).

### Cell colony formation assay

The transfected HCCLM3 and Huh7 cells (1 × 10^2^) were seeded in a cell culture dish and maintained for 9 days. The medium was replaced every 3–4 days. The cells were fixed with ethanol (75%) for 2 h and then stained with crystal violet (0.2%, KeyGen, Jiangsu, China) for 2 h. The number of cells colonies (> 50 cells/colony) was counted and photographed by using the light microscope (Olympus, Tokyo, Japan).

### Flow cytometry assay

The cell cycle distribution was assessed with propidium iodide (PI) cytometry assay. In short, the transfected HCCLM3 and Huh7 cells were cultured for 48 h. Then, the cells were harvested and fixed with ethanol (70%) at − 20 °C for overnight. Thereafter, the cells were washed with phosphate buffer solution (PBS) and then stained with the PI/RNase solution (Sigma). The cell cycle distribution was assessed with the FACScan flow cytometry (BD Biosciences, Bedford, MA, USA).

### Wound healing assay

The migration ability of the transfected HCCLM3 and Huh7 cells was assessed with the scratch test. After transfection for 48 h, HCCLM3 and Huh7 cell monolayers (with the confluency of 90%) were scratched via a pipette tip (200 μL). Thereafter, the cells were washed with PBS and then cultured in RPMI 1640 medium (with or without FBS). Wounds were observed at 0 h, 12, or 24 h, respectively. The images were obtained with the light microscope (Olympus).

### Transwell assay

The invasion capacity of transfected HCCLM3 and Huh7 cells was evaluated using the transwell chamber (8 μm, BD Biosciences) with matrigel matrix (BD Biosciences). After culture for 24 h, the transfected HCCLM3 and Huh7 cells were (3 × 10^4^ cells) were seeded to the top chamber with RPMI 1640 medium (without FBS). And the RPMI 1640 medium (with 10% FBS) was supplemented into the lower of the transwell chamber as a chemoattractant and cultured for 24 h. After removing the cells on the upper surface of the membrane with a cotton swab, the cells on the lower surface of the membrane were fixed with methanol (100%) and stained with crystal violet (0.25%, Sigma). The invaded cells were counted via a light microscope (Olympus).

### Western blot analysis

Specimens, HCC xenograft tissues, and cells were lysed in lysis buffer (Beyotime, Shanghai, China). Western blot analysis was executed as previously described [29]. Total protein concentration was evaluated via the Bicinchoninic Acid Protein Assay Kit (Beyotime). Protein bands were visualized by the ImmunoStar LD (Wako Pure Chemical, Osaka, Japan). The primary antibodies used were presented as follows: anti-Cyclin D1 (ab134175, 1:1000), anti-matrix metalloproteinase-2 (MMP2) (ab92536, 1:1000), anti-matrix metalloproteinase-9 (MMP9) (ab76003, 1:1000), anti-SMAD6 (ab80049, 1:500), anti-proliferating cell nuclear antigen (PCNA) (ab92552, 1:1000), and anti-GAPDH (ab128915, 1:5000). The goat anti-rabbit (ab97051, 1:10,000) immunoglobulin G (IgG) used as the secondary antibody. Also, GAPDH was regarded as a loading control. All antibodies were bought from Abcam (Cambridge, MA, USA).

### Dual-luciferase reporter assay

The binding sites of miR-326 in hsa_circ_0000517 were predicted with the Circular RNA Interactome and Starbase databases. The sequence of hsa_circ_0000517 (possessed binding sites for miR-326) was inserted into the pGL3-control vector (Promega, Madison, WI, USA) to construct the luciferase reporters with wild type (wt) hsa_circ_0000517. And the luciferase reporters with the mutant (mut) hsa_circ_0000517 (within the binding sites to miR-326) were also established via using the same way. The binding sites of SMAD6 in miR-326 were predicted with the targetscan database. The luciferase reporters containing SMAD6-wt 3′Untranslated Regions (UTR) or SMAD6-mut 3′UTR were constructed using the same method. HCC cells were co-transfected luciferase reporters and NC or miR-326 using Lipofectamine 3000 reagent. The luciferase intensities of luciferase reporters in HCC cells were determined with the dual-luciferase reporter assay kit (Promega).

### RNA immunoprecipitation (RIP) assay

The relationship between hsa_circ_0000517 or SMAD6 and miR-326 was confirmed through the Magna RIP kit (Millipore, Bedford, MA, USA). HCC cells were lysed by using the RIP lysis buffer. The cell lysates were incubated with the RIP buffer containing magnetic beads conjugated with anti-Ago2 or anti-IgG antibodies (Millipore). Next, the magnetic beads were incubated with proteinase K (Sigma), and the total RNA was isolated using the TRIzol reagent (Life Technologies). QRT-PCR was employed to assess the abundance of hsa_circ_0000517, SMAD6, and miR-326.

### Xenograft assay

10 BALB/c nude mice (athymic, 5-week-old, 17–18 g) were purchased from Shanghai Experimental Animal Center (Shanghai, China) and kept under specific-pathogen-free conductions. The animal experiment was ratified by the Animal Ethics Committee of the First Affiliated Hospital of Zhengzhou University. Huh7 cells with sh-NC or stable lentivirus-mediated sh-hsa_circ_0000517 (GenePharma) were subcutaneously injected into the dorsal side of the nude mice. The tumor volume was measured once a week from the day of injection and calculated by the equation: Volume = (length × width^2^)/2. The mice were euthanized on day 35 to obtain the tumor tissues for subsequent analysis.

### Statistical analysis

Statistical analysis was conducted via 19.0 (SPSS, Chicago, IL, USA). Differences with *P* < 0.05 were statistically. Data were exhibited as mean ± standard deviation. Chi square test was used to evaluate the correlation between hsa_circ_0000517 expression and clinicopathological parameters. The experiments in vitro were performed in triplicate. Statistical significance was evaluated by Student’s *t* test (the differences between two groups) or one-way variance analysis (ANOVA) (the differences among more groups). The correlation was determined with Pearson’s correlation analysis. The survival rate was analyzed through the Kaplan–Meier curves and the log-rank test.

## Results

### High hsa_circ_0000517 expression in HCC tissues and cells was associated with poor prognosis

At outset, we examined the expression of hsa_circ_0000517 in 50 paired HCC tissues and adjoining normal tissues via qRT-PCR. We observed that hsa_circ_0000517 expression was overtly increased in HCC tissues with respect to the adjoining normal tissues (Fig. 1a). Furthermore, high hsa_circ_0000517 expression was associated with tumor size (*P *< 0.0001), TNM state (*P *= 0.0016), and lymph node metastasis (*P *= 0.0039) (Table 1). Based on the median of patients with HCC, we divided HCC patients into high hsa_circ_0000517 expression group and low hsa_circ_0000517 expression group (Fig. 1b). Moreover, the survival time of HCC patients with the high expression of hsa_circ_0000517 was shorter than those with the decrease expression of hsa_circ_0000517 (Fig. 1c). We also analyzed the characteristic of hsa_circ_0000517 in HCC cells. And hsa_circ_0000517 was resistant to RNase R compared to the liner gene RPPH1 (Fig. 1d). Consistently, the expression of hsa_circ_0000517 was signally elevated in HCC cells (HCCLM3, Huh7, and MHCC97-H) in contrast to the THLE-2 cells, and hsa_circ_0000517 expression was higher in HCCLM3 and Huh7 cells (Fig. 1e). These data manifested that elevated hsa_circ_0000517 expression might be connected with HCC advancement.

**Fig. 1:** Expression level of hsa_circ_0000517 in HCC tissues and cells. **a** QRT-PCR was conducted to detect hsa_circ_0000517 expression in 50 paired HCC tissues and adjoining normal tissues. **b** High hsa_circ_0000517 expression and low hsa_circ_0000517 expression were divided according to the median of patients with HCC. **c** Kaplan–Meier curves and log-rank test were employed to determine the survival time of HCC patients with high hsa_circ_0000517 expression and low hsa_circ_0000517 expression. **d** QRT-PCR was employed to assess the resistance of hsa_circ_0000517 and RPPH1 to RNase R. **e** QRT-PCR was performed to evaluate hsa_circ_0000517 expression in HCCLM3, Huh7, and MHCC97-H, and THLE-2 cells. *P < 0.05

### Silence of hsa_circ_0000517 repressed cell proliferation, colony formation, migration, and invasion, and induced cell cycle arrest in HCC cells

In view of the enhancement of hsa_circ_0000517 in HCC tissues and cells, we investigated the role of hsa_circ_0000517 in HCC via loss-of-function experiments. We designed two siRNA targeting hsa_circ_0000517 (si-hsa_circ_0000517#1 and si-hsa_circ_0000517#2) and results of qRT-PCR exhibited that hsa_circ_0000517 expression was markedly decreased in HCCLM3 and Huh7 cells transfected with si-hsa_circ_0000517#1 and si-hsa_circ_0000517#2 (Fig. 2a). CCK-8 assay displayed that cell proliferation was apparently suppressed in hsa_circ_0000517-silenced HCCLM3 and Huh7 cells (Fig. 2b). Also, cell colony formation assay manifested that hsa_circ_0000517 inhibition evidently repressed cell colony formation capacity in HCCLM3 and Huh7 cells (Fig. 2c). Moreover, the cell percentage in the G1 stage of cell cycle was notably increased in HCCLM3 and Huh7 cells (Fig. 2d). And hsa_circ_0000517 silencing reduced the levels of p21 and enhanced the levels of C-caspase 3 in HCCLM3 and Huh7 cells (Additional file 1: Fig. S1). Wound healing assay presented that the migratory rate of HCCLM3 and Huh7 cells was conspicuously decreased after hsa_circ_0000517 inhibition (Fig. 2e). Likewise, regardless of the presence of FBS, the migratory rate of HCCLM3 and Huh7 cells was reduced after hsa_circ_0000517 knockdown, indicating that hsa_circ_0000517 silencing could decrease the migration of HCCLM3 and Huh7 cells (Additional file 2: Fig. S2). As expected, transwell assay also disclosed that reduced hsa_circ_0000517 expression impeded cell invasion capacity in HCCLM3 and Huh7 cells (Fig. 2f). Furthermore, Cyclin D1, MMP2, and MMP9 were down-regulated in hsa_circ_0000517-suppressed HCCLM3 and Huh7 cells (Fig. 2g). In all, these results demonstrated that hsa_circ_0000517 silencing repressed the malignant behaviors of HCC cells.

**Fig. 2:** Effects of hsa_circ_0000517 down-regulation on proliferation, colony formation, cell cycle, migration, and invasion of HCC cells. **a**–**g** HCCLM3, Huh7 cells were transfected with si-hsa_circ_0000517#1, si-hsa_circ_0000517#2, or si-NC. **a** The expression of hsa_circ_0000517 in HCCLM3 and Huh7 cells was analyzed by qRT-PCR. **b**–**f** The proliferation, colony formation, cell cycle, migration, and invasion of HCCLM3 and Huh7 cells were analyzed via CCK-8 (**b**), colony formation (**c**), flow cytometry (**d**), wound healing (**e**), or transwell assays (**f**). **g** The protein levels of Cyclin D1, MMP2, and MMP9 in HCCLM3 and Huh7 cells were detected with western blot analysis. *P < 0.05

### Hsa_circ_0000517 was identified as a ceRNA for miR-326

Then, we further explored the molecular mechanism of hsa_circ_0000517 in HCC. We discovered that miR-1296-5p, miR-326, and miR-330-5p might be potential targets for hsa_circ_0000517 through Starbase and Circular RNA Interactome databases (Fig. 3a). And miR-326 expression was higher than that of miR-1296-5p and miR-330-5p in hsa_circ_000051-sileced HCCLM3 and Huh7 cells (Additional file 3: Fig. S3). The binding sites of hsa_circ_0000517 in miR-326 and its mutant sites were displayed in Fig. 3b. Moreover, we observed that miR-326 expression was remarkably decreased in HCC tissues in comparison to the adjoining normal tissues (Fig. 3c). And miR-326 was down-regulated in HCCLM3, Huh7, and MHCC97-H cells than that in the THLE-2 cells (Fig. 3d). The correlation analysis revealed that the expression of hsa_circ_0000517 and miR-326 in HCC tissues had negative correlation (Fig. 3e). We observed that hsa_circ_0000517 was overtly increased in HCCLM3 and Huh7 cells after hsa_circ_0000517 transfection (Additional file 4: Fig. S4A). Also, miR-326 expression was distinctly restrained by hsa_circ_0000517 overexpression and was accelerated by hsa_circ_0000517 silencing in HCCLM3 and Huh7 cells (Fig. 3f). And miR-326 expression was enhanced after miR-326 transfection and was reduced by transfecting with anti-miR-326 in HCCLM3 and Huh7 cells (Additional file 4: Fig. S4B). Besides, dual-luciferase reporter assay manifested that miR-326 enhancement inhibited the luciferase intensity of the luciferase reporter with hsa_circ_0000517-wt in HCCLM3 and Huh7 cells, while there was no visible difference in hsa_circ_0000517-mut luciferase reporters (Fig. 3g). RIP assay exhibited that hsa_circ_0000517 and miR-326 were dramatically enriched in Ago2-containing micro-ribonucleoprotein complexes, indicating that Ago2 protein bound to hsa_circ_0000517 and miR-326 in HCCLM3 and Huh7 cells (Fig. 3h). Taken together, these findings revealed that hsa_circ_0000517 served as a ceRNA for miR-326 in HCC.

**Fig. 3:** MiR-326 acted as a target for hsa_circ_0000517 in HCC. **a** Both Starbase and Circular RNA Interactome databases displayed that miR-1296-5p, miR-326, and miR-330-5p might be potential targets for hsa_circ_0000517. **b** The binding sites of hsa_circ_0000517 in miR-326 were showed. **c**, **d** QRT-PCR was employed to detect miR-326 expression in HCC tissues and cells. **e** The correlation between hsa_circ_0000517 and miR-326 in HCC tissues was revealed via Pearson’s correlation analysis. **f** Effect of hsa_circ_0000517 on miR-326 expression of HCCLM3 and Huh7 cells was determined by qRT-PCR. **g** The luciferase intensity in HCCLM3 and Huh7 cells co-transfected luciferase reporters containing hsa_circ_0000517-wt or hsa_circ_0000517-mut and miR-326 or NC was determined through dual-luciferase reporter assay. **h** The relationship between hsa_circ_0000517 and miR-326 was further verified via RIP assay. *P < 0.05

### MiR-326 silencing overturned hsa_circ_0000517 inhibition-mediated effects on proliferation, colony formation, cell cycle, migration, and invasion of HCC cells

Given that miR-326 acted as a target for hsa_circ_0000517 in HCC, we further checked on whether hsa_circ_0000517 exerted its role through miR-326. QRT-PCR revealed that the elevation of miR-326 in HCCLM3 and Huh7 cells caused by hsa_circ_0000517 inhibition was reversed by anti-miR-326 introduction (Fig. 4a). Moreover, the inhibitory impacts of hsa_circ_0000517 depletion on proliferation and colony formation of HCCLM3 and Huh7 cells were abolished by miR-326 down-regulation (Fig. 4b, c). Furthermore, miR-326 inhibition reversed the repression of cell cycle of HCCLM3 and Huh7 cells induced by hsa_circ_0000517 down-regulation (Fig. 4d). Also, decreased miR-326 expression recovered the suppressive effects on migration and invasion of HCCLM3 and Huh7 cells mediated by hsa_circ_0000517 silencing (Fig. 4e, f). Moreover, the down-regulation of Cyclin D1, MMP2, and MMP9 in hsa_circ_0000517-constrained HCCLM3 and Huh7 cells were restored by miR-326 repression (Fig. 4g). Together, these results indicated that hsa_circ_0000517 silencing repressed HCC progression via miR-326.

**Fig. 4:** Hsa_circ_0000517 played its role in HCC via miR-326. **a** The si-NC, si-hsa_circ_0000517#1, si-hsa_circ_0000517#1 + anti-NC, or si-hsa_circ_0000517#1 + anti-miR-326 was transfected into HCCLM3 and Huh7 cells, respectively. **a** The expression of miR-326 in HCCLM3 and Huh7 cells was analyzed through qRT-PCR. **b**–**f** The proliferation, colony formation, cell cycle, migration, and invasion of HCCLM3 and Huh7 cells was evaluated with CCK-8 (**b**), colony formation (**c**), flow cytometry (**d**), wound healing (**e**), or transwell assays (**f**). **g**, **h** Protein levels of Cyclin D1, MMP2, and MMP9 in HCCLM3 and Huh7 cells were examined via western blot analysis. *P < 0.05

### SMAD6 acted as a target for miR-326

Next, we explored the downstream target for miR-326 in HCC via targetscan database. The 3′UTR of SMAD6 possessed the possible binding sites for miR-326, as exhibited in Fig. 5a. The levels of SMAD6 mRNA and protein were obviously increased in HCC tissues compared to the adjoining normal tissues (Fig. 5b, c). Congruously, SMAD6 protein level was up-regulated in HCC cells (Fig. 5d). The levels of SMAD6 mRNA were enhanced by transfecting with SMAD6 and were decreased by transfecting with si-SMAD6 in HCCLM3 and Huh7 cells (Additional file 4: Fig. S4C). We also detected the levels of pSMAD1/5/8 in HCCLM3 and Huh7 cells. The results exhibited that SMAD6 knockdown increased the levels of pSMAD1/5/8 in HCCLM3 and Huh7 cells. These results indicated that SMAD6 silencing could activate the SMAD signaling (Additional file 5: Fig. S5). Moreover, the expression of SMAD6 in HCC tissues had a positive correlation with hsa_circ_0000517 and negative correlation with miR-326 (Fig. 5e, f). Also, enhanced miR-326 expression constrained SMAD6 protein levels in HCCLM3 and Huh7 cells, while this impact was recovered by hsa_circ_0000517 overexpression (Fig. 5g). Additionally, dual-luciferase reporter assay disclosed that the luciferase activity was overtly repressed in HCCLM3 and Huh7 cells co-transfected with miR-326 and luciferase reporters with SMAD6-wt, while the luciferase activity in luciferase reporters with SMAD6-mut did not change (Fig. 5h). RIP assay suggested that miR-326 and SMAD6 were gathered in Ago2-harboring miRNA ribonucleoprotein complexes compared the control group (Fig. 5i). These results indicated that SMAD6 was a target for miR-326 in HCC.

**Fig. 5:** MiR-326 targeted SMAD6 in HCC cells. **a** The predicted binding sites between 3′ UTR of SMAD6 and miR-326 were predicted with targetscan database. **b**, **c** The levels of SMAD6 mRNA and protein in HCC tissues were detected via qRT-PCR or western blot analysis. **d** The level of SMAD6 protein in HCC cells was examined via western blot analysis. **e**, **f** The correlation between SMAD6 and hsa_circ_0000517 or miR-326 in HCC tissues was assessed with Pearson’s correlation analysis. **g** Effect of hsa_circ_0000517 overexpression on SMAD6 protein levels of miR-326-enhanced HCCLM3 and Huh7 cells was analyzed through western blot analysis. **h** Dual-luciferase reporter assay was executed to determine the luciferase intensity of the luciferase reporters containing SMAD6-wt or SMAD6-mut in HCCLM3 and Huh7 cells transfected with miR-326 or NC. **i** RIP assay was conducted to assess the miR-326 and SMAD6 enrichment in immunoprecipitates in HCCLM3 and Huh7 cells. *P < 0.05

### SMAD6 elevation abrogated miR-326 overexpression-mediated impacts on proliferation, colony formation, cell cycle, migration, and invasion of HCC cells

Considering that miR-326 targeted SMAD6 in HCC cells, we further verified the interaction between miR-326 and SMAD6 in HCC cells. We discovered that SMAD6 overexpression partly reversed the inhibitory effect of miR-326 mimics on the levels of SMAD6 protein of HCCLM3 and Huh7 cells (Fig. 6a). Moreover, SMAD6 overexpression overturned the repressive effects on proliferation, colony formation, and cell cycle progression of HCCLM3 and Huh7 cells mediated by miR-326 up-regulation (Fig. 6b–d). Also, the inhibition of migration and invasion of HCCLM3 and Huh7 cells induced by miR-326 enhancement was restored by SMAD6 elevation (Fig. 6e, F). In addition, the protein levels of Cyclin D1, MMP2, and MMP9 in miR-326-elevated HCCLM3 and Huh7 cells were repressed, while this suppression was abolished by SMAD6 augmentation (Fig. 6g, h). Collectively, these results indicated that miR-326 played its role via targeting SMAD6 in HCC cells.

**Fig. 6:** MiR-326 exerted its role through SMAD6 in HCC cells. **a** Western blot analysis was conducted to assess the influence of SMAD6 overexpression on SMAD6 protein levels of miR-326-elevated HCCLM3 and Huh7 cells. **b**–**f** Impacts of SMAD6 augmentation on miR-326 enhancement-mediated proliferation, colony formation, cell cycle, migration, and invasion of HCCLM3 and Huh7 cells were determined with CCK-8 (**b**), colony formation (**c**), flow cytometry (**d**), wound healing (**e**), or transwell assays (**f**). **g**, **h** Effects of SMAD6 overexpression on the levels of Cyclin D1, MMP2, and MMP9 of miR-326-elevated HCCLM3 and Huh7 cells were evaluated via western blot analysis. *P < 0.05

### Hsa_circ_0000517 down-regulation constrained HCC growth in vivo

In view of the repressive effects of hsa_circ_0000517 silencing on cell malignant behaviors in vitro, we further verified the role of hsa_circ_0000517 down-regulation on tumor growth in vivo via xenograft assay. We observed that tumor volume and weight were prominently repressed in the sh-hsa_circ_0000517 group compared to the control group (Fig. 7a, b). Furthermore, hsa_circ_0000517 expression was evidently repressed in tumor tissues of the sh-hsa_circ_0000517 group in comparison with the sh-NC group, while the expression of miR-326 was visibly elevated (Fig. 7c, d). Besides, PCNA and SMAD6 protein levels were also distinctly down-regulated in tumor tissues of the sh-hsa_circ_0000517 group (Fig. 7e). In sum, these data indicated that hsa_circ_0000517 repletion could repress HCC growth in vivo.

**Fig. 7:** Depletion of hsa_circ_0000517 repressed HCC growth in vivo. **a** Tumor volumes were measured once a week from the day of injection. **b** Tumor weight in the sh-hsa_circ_0000517 and sh-NC groups was assessed on day 35. **c**, **d** The expression of hsa_circ_0000517 and miR-326 in tumor tissues of the sh-hsa_circ_0000517 and sh-NC groups was detected with qRT-PCR. **e** Protein levels of PCNA and SMAD6 in tumor tissues of the sh-hsa_circ_0000517 and sh-NC groups were examined by western blot analysis. *P < 0.05

## Discussion

Recently, more and more cancer-associated circRNAs were revealed, and some of them were connected with HCC tumorigenesis and advancement [12]. For instance, circRNA circMTO1 constrained HCC progression via sponging miR-9 [30]. CircRNA has_circ_000145 suppressed metastasis and growth of HCC by up-regulating TIMP3 via miR-17-3p and miR-181-5p [31]. Also, circRNA has_circ_104718 increased TXNDC5 expression via targeting miR-218-5p, which accelerated cell apoptosis and inhibited cell invasion, proliferation, and migration in HCC cells [32]. Herein, HCC patients with high hsa_circ_0000517 expression had a lower survival rate. Moreover, hsa_circ_0000517 reduction repressed tumor growth in vivo and suppressed proliferation, colony formation, cell cycle progression, migration, and invasion of HCC cells in vitro. Wang et al. also disclosed that high hsa_circ_0000517 expression could predict the adverse prognosis of HCC [13]. Hence, we could conclude that hsa_circ_0000517 acted as an oncogene in HCC.

Increasing researches manifested that circRNAs were in involved in the progression of diverse cancers by acting as a ceRNA for miRNAs [30, 32, 33]. MiR-326 was demonstrated to be a suppressor in various cancers. In lung cancer, long non-coding RNA (lncRNA) HOTAIR regulated the miR-326/PHOX2A axis, which repressed cell apoptosis and promoted cell migration, proliferation, and cell cycle progression [18]. Moreover, forced miR-326 expression induced cell apoptosis and cycle arrest, and curbed cell colony formation, invasion, migration, and proliferation in prostatic carcinoma cells [34]. Another one reporter revealed that miR-326 was up-regulated by has_circ_0000515 inhibition in cervical cancer cells, which could facilitate cell apoptosis, autophagy, and repressed cell invasion and proliferation [35]. Besides, miR-326 could be repressed by lncRNA H19, lncRNA SNHG3, or circRNA circASAP1, respectively, which could contribute to HCC progression [36–38]. Moreover, miR-326 could act as a promising biomarker for prognosis evaluation and diagnosis, and it could lead to the development of new cancer therapies [39]. In our study, miR-326 acted as a target for hsa_circ_0000517. Moreover, the inhibition of miR-326 reversed hsa_circ_0000517 depletion-mediated effects on the malignant behaviors of HCC cells. Hence, it is possible that miR-326 serve as a new target for HCC therapy.

Additionally, we found that SMAD6 was a downstream target for miR-326. SMAD6 was regulated by hsa_circ_0000517 through miR-326. Moreover, the overexpression of SMAD6 abolished the repressive impacts of miR-326 up-regulation on proliferation, colony formation, cell cycle, migration, and invasion of HCC cells. A study revealed that BRG1 promoted HCC cell proliferation and predicted HCC recurrence through up-regulating SMAD6 [28]. Another study demonstrated that galangin inhibited the proliferation of HepG2 cells via activation of the TGF-β/SMAD pathway [40]. In consequence, we concluded that hsa_circ_0000517 could regulate HCC progression via the miR-326/SMAD6 axis (Fig. 8).

**Fig. 8:** Schematic diagram of the mechanism of hsa_circ_0000517 involved in HCC advancement. Hsa_circ_0000517 promoted HCC progression via up-regulating SMAD6 via miR-326

## Conclusion

In all, hsa_circ_0000517 acted as an oncogene in HCC. Furthermore, hsa_circ_0000517 silencing repressed HCC progression through reducing SMAD6 expression via targeting miR-326. The research suggested that hsa_circ_0000517 served as a promising prognostic marker and therapeutic target for HCC.

## Supplementary information

**Additional file****1****: Fig. S2** Effect of hsa_circ_0000517 inhibition on p21 and C-caspase 3 levels of HCC cells. (A and B) The levels of p21 and C-caspase 3 in HCCLM3 and Huh7 cells transfected with si-hsa_circ_0000517#1, si-hsa_circ_0000517#2, or si-NC were measured with western blot analysis. *P < 0.05.

**Additional file****2****: Fig. S5** Impact of hsa_circ_0000517 silencing on the migration of HCC cells. (A and B) Wound healing assay was performed to assess the migration of HCCLM3 and Huh7 cells with or without FBS. *P < 0.05.

**Additional file****3****: Fig. S4** Influence of hsa_circ_0000517 knockdown on miRNAs expression of HCC cells. (A and B) The expression of miR-1296-5p, mire-326, and miR-330-5p in HCCLM3 and Huh7 cells transfected with si-hsa_circ_0000517#1 or si-NC was evaluated via qRT-PCR. *P < 0.05.

**Additional file****4****: Fig. S1** Efficiency of cell transfection of plasmids and oligonucleotides. (A-C) The levels of hsa_circ_0000517, miR-326, or SMAD6 in HCCLM3 and Huh7 cells transfected with circ-NC, hsa_circ_0000517, NC, miR-326, anti-NC, anti-miR-326, vector, SMAD6, si-NC, or si-SMAD6 were assessed by qRT-PCR. *P < 0.05.

**Additional file****5****: Fig. S3** Effect of SMAD6 knockdown on SMAD signaling of HCC cells. (A and B) The levels of pSMAD1/5/8 in HCCLM3 and Huh7 cells were examined with western blot analysis. *P < 0.05.

## Data Availability

All data generated or analysed during this study are included in this published Article.

## Abbreviations

HCC: Hepatocellular carcinoma
hsa_circ_0000517: Circular RNA hsa_circ_0000517
SMAD6: SMAD family member 6
CCK-8: Cell Counting Kit-8
MMP2: Matrix metalloproteinase-2
MMP9: Matrix metalloproteinase-9
PCNA: Proliferating cell nuclear antigen
RIP: RNA immunoprecipitation
